# A Review of Carcinomas Arising in the Head and Neck Region in HIV-Positive Patients

**DOI:** 10.4061/2011/469150

**Published:** 2011-05-10

**Authors:** Bibianna Purgina, Liron Pantanowitz, Raja R. Seethala

**Affiliations:** Department of Pathology, Presbyterian-Shadyside University Hospital, University of Pittsburgh Medical Center, Pittsburgh, PA 15213, USA

## Abstract

The majority of malignancies arising in the head and neck among patients with AIDS are Kaposi sarcoma and non-Hodgkin lymphoma. Patients with HIV/AIDS are also at increased risk of developing several carcinomas of the head and neck. This paper focuses on these less common, albeit important, carcinomas. An English language literature search identified numerous population-based studies evaluating carcinomas in the head and neck of HIV-positive patients. Published results indicate that patients with HIV/AIDS are at an increased risk of developing mucosal squamous cell carcinoma, nasopharyngeal carcinoma, lymphoepithelial carcinoma of the salivary gland, and Merkel cell carcinoma in this anatomic region. Data also suggest that HIV-positive patients with these cancers present at a younger age, with more aggressive disease and worse prognosis compared to HIV-negative patients. Treatment involves surgical resection with or without radiation therapy and chemotherapy for locally advanced and metastatic disease. AIDS patients, however, are more likely to suffer radiation treatment complications. Highly active antiretroviral therapy (HAART) has not altered the incidence of these malignancies.

## 1. Introduction

An increased rate of neoplastic disease is a well-established phenomenon in patients with human immunodeficiency virus (HIV) and acquired immunodeficiency syndrome (AIDS). In contrast to squamous cell carcinoma (SCC), which is by far the most common head and neck malignancy in HIV-negative patients, the majority of malignancies arising in the head and neck among patients with AIDS are the virally-induced AIDS-defining cancers (ADCs): Kaposi sarcoma (KS) and non-Hodgkin lymphoma (NHL), most commonly large B-cell and plasmablastic lymphomas. However, as the HIV pandemic persists and more people are living with chronic HIV infection, the spectrum of non-AIDS defining cancers (NADCs) seems to be increasing. The incidence of NADC in the head and neck in patients with HIV and AIDS is similalry increasing, including squamous cell carcinoma (SCC), lymphoepithelial carcinoma (LEC) of the salivary gland, nasopharyngeal carcinoma (NPC) and Merkel cell carcinoma (MCC).

These aforementioned epithelial malignancies all demonstrate a relationship to oncogenic viruses including Human Papilloma virus (HPV), Epstein-Barr virus (EBV) or Merkel cell polyoma virus (MCV). Since the oropharynx and respiratory tract is a common site for the persistence and transmission of these oncogenic viruses, it is possible that patients with HIV/AIDS may be at increased risk of developing head and neck cancers compared to the general population. However, confounding etiologic factors also exist since HIV-positive individuals generally have higher smoking rates and greater alcohol consumption, both independent risk factors for head and neck neoplasms, compared to HIV-negative individuals [1–4]. This paper presents the epidemiology, etiology, clinical features, pathologic findings, prognosis and management of the most commonly reported epithelial NADC arising in the head and neck region of patients with HIV/AIDS.

## 2. Methods

A literature review was performed using PubMed as well as cited references within previously published articles and textbooks for all published studies related to the incidence of head and neck epithelial carcinomas (non-KS, non-NHL) in patients with documented HIV infection. The study was confined to articles in English. An attempt was made to avoid duplicate cases published in the literature. Standardized incidence ratios (SIRs) and/or relative risks (RR), along with 95% confidence interval (95% CI)-were extracted and tabulated.

## 3. Epidemiology

In the USA, approximately 36,540 individuals in the general population are diagnosed yearly with head and neck malignancies, and approximately 7,880 die of their illness [5]. Epithelial malignancies of the head and neck are most common in men over the age of 50 years and have a strong association with cigarette smoking and alcohol consumption. They are also associated with the oncogenic viruses, EBV and HPV, typically in the nasopharynx and oropharynx, respectively. In patients with HIV, a statistically significant increased risk has been reported for salivary gland LEC and NPC as well as SCC of the lip, oropharynx, and conjunctiva [4, 6–14]. Even though the results have been variable [6, 8, 11, 13, 15–17], it appears that patients with HIV present at a younger age, with more aggressive disease and worse prognosis compared to their HIV-negative counterparts [10, 11, 18–20].

## 4. Etiology

### 4.1. Immunosuppression

In comparison to patients with HIV/AIDS, large population-based studies in immunosuppressed transplant recipients have demonstrated a wider range of malignancies that may be associated with immunodeficiency. A meta-analysis comparing both HIV-positive and HIV-negative immune suppressed patient groups showed that an extensive range of malignancies occurred at an increased incidence in both populations and that the pattern of increased risk was similar [21]. Many of these cancers are associated with a known infectious entity including HPV, EBV, Human Polyoma virus, Hepatitis B and C and others, and suggest that the range of infection-related malignancies seen in immunodeficient patients is much wider than previously described. Of the HPV-related malignancies, SCC of the lip, oral cavity, pharynx and conjunctiva showed an increased incidence in HIV-negative and HIV-positive immunosuppressed patient populations. NPC seems to occur more commonly in patients with HIV/AIDS, compared to transplant recipients. The SIR for NPC arising in patients with HIV/AIDS was 2.90 (95% CI 1.8–4.66) in people with HIV/AIDS. Only a single case of NPC was reported in a transplant recipient [21]. It is important to keep in mind that cigarette smoking is different in these two populations, with renal transplant patients' cigarette smoking rates being similar to the general population [22] and more than double those of patients with HIV/AIDS [2]. However, a meta-analysis of SIRs for tobacco-related cancers were not found to be consistently higher in cohorts with HIV/AIDS [21].

In a large cohort study using nation-wide linkage data, Grulich et al. [13] showed that patients with AIDS demonstrate increased rates of several NADCs, whereas patients with HIV and mild immunodeficiency were only at increased risk of anal cancer. Other cancers were seen only later in the course of HIV-infection. These findings suggest that HIV-positive patients with only mild immunodeficiency may not be at an increased risk of NADCs. One study suggests that there may be increased risk of oropharyngeal carcinoma with increasing severity of AIDS-related immunodeficiency [10].

Since the introduction of highly active antiretroviral therapy (HAART), most HIV-positive patients are now living with only mild to moderate degrees of immunodeficiency for extended periods, and patients with AIDS now represent an increasing minority. Thus, it is becoming increasingly important to study the association between the degree and duration of immunodeficiency and the risk of cancer. In transplant recipients with prolonged immunosuppression, there is a striking increased risk of HPV-related carcinomas suggesting that even modest immunosuppression, if present for a long period, can increase the risk of these cancers [22]. Similar studies in mild-to-moderately immunodeficient HIV-positive patients receiving HAART are needed.

### 4.2. Oncogenic Viruses

The oropharyngeal compartment is central to the persistence and transmission of both EBV and HPV. Studies have shown that EBV and HPV are more commonly detected in the oral mucosa of HIV-positive patients compared to HIV-negative patients [23, 24]. Ammatuna et al. [23] detected EBV and HPV in the oral mucosa of 17% and 3% of HIV-negative patients, respectively, and 42% and 7% of HIV-positive patients. Kreimer et al. [24] found similar results examining the prevalence of oral high-risk HPV infection among HIV-positive and HIV-negative patients (13.7% in HIV-positive patients compared with 4.5% in HIV-negative patients).

The association between HIV and HPV in the context of cervical cancer is well-established and it has been demonstrated that the development and detection of cervical squamous intraepithelial lesion (SIL) are directly proportional to the severity of HIV-induced immunosuppression, measured by low CD4 counts and high HIV viral loads [25, 26]. HPV, most commonly subtype 16, is responsible for some oral cavity carcinomas, more than 60% of oropharyngeal carcinomas, and approximately 90% of tonsillar carcinomas [27–31]. There are many other studies linking HPV infection to SCC of the larynx and conjunctiva [32–34], and this may also explain the increased risk of these carcinomas in immunodeficient patients [21, 27]. Some studies have shown that HPV-containing cancers of the head and neck lack p53 mutations, unlike the HPV-negative cancers at these sites [35–37]. It is well established that the E6 protein of HPV 16 inactivates p53 protein, an important component of the cell cycle, which leads to increased rates of mutagenesis. Thus, the pathogenesis of HPV-associated SCC of the head and neck in patients with HIV/AIDS includes increased proliferation of neoplastic cells caused by viral interference with tumor suppressor genes (p53 and retinoblastoma) from viral proteins generated by both HIV and HPV [35–39]. While AIDS patients have been shown to be at increased risk of developing HPV-associated oropharyngeal carcinomas (SIR 1.6, 95% CI 1.2–2.1), it is possible that confounding factors such as increased cigarette smoking rates may account for some of this increased risk [10].

Following primary infection with EBV, this herpes virus may undergo active lytic replication releasing viral progeny or may initiate active latency in which one of three restricted gene expression programs is initiated. Type I latency with expression of only EBER (EBV early RNAs) and EBNA-1 (EBV nuclear antigens) is typical of Burkitt lymphoma. Type II latency demonstrates the expression of EBER, EBNA-1, and latent membrane proteins (LMPs) and is seen in nasopharyngeal carcinoma. Both latency patterns I and II have been identified in LEC of the salivary gland. EBV is also associated with a variety of other epithelial carcinomas including LEC of the stomach, lung and thymus [35]. EBV has also been implicated in the chronic inflammatory condition known as HIV-related sialadenitis. Chronic sialadenitis is also known to be a risk for salivary gland carcinoma [35]. It has been suggested that altered immunity may be important for the development of EBV-related salivary gland carcinomas since they have also been described in patients with chronic autoimmune disease [40].

MCC also commonly affects immunocompromised patients, suggesting infectious etiology. With great excitement, the association with MCV (also referred to as MCPyV) was recently established [41]. In MCC, the viral DNA is integrated into the tumor genome in a clonal manner [41]. This suggests that infection and integration of the MCV occurs prior to the clonal expansion of the tumor cells and implicates this virus in the pathogenesis of MCC. Once inserted into the host DNA, viral T antigen is expressed as large T and small T antigens. These T antigens in turn alter the behavior of tumor suppressor and cell cycle regulatory proteins such as Rb, p53, protein phosphatase 2A, and Bub1 [42]. Other risk factors including increased exposure to ultraviolet (UV) and ionizing radiation may also be involved in T-antigen mutations. Although MCV may be present in cutaneous MCC, it has not been found in similar mucosal high-grade neuroendocrine carcinomas [43]. On the other hand, common warts can be positive for MCV in immunosuppressed individuals [44], but not SCC or basal cell carcinoma (BCC) of the skin [45].

### 4.3. Nonviral Cofactors

There is a strong association between head and neck SCC and cigarette smoking and heavy alcohol consumption. In fact, these two risk factors are strongly synergistic and may account for approximately 75% of these SCCs [46]. There are numerous studies demonstrating that smoking is more common in HIV-positive persons [1–4, 47], which may explain the increased rates of head and neck carcinomas, especially SCC in this population. However, it is unlikely that cigarette smoking alone can explain the statistically significant increased rates of head and neck SCC observed arising in HIV infected patients significantly younger than their HIV-negative counterparts [10, 11, 14, 18, 19, 48]. In a prospective study out of France, 11% of deaths in HIV positive patients resulted from cancers not caused by hepatitis and unrelated to HIV, and in these cases, smoking and excess alcohol consumption were recorded in 72% and 27% of these cancer deaths respectively [49]. In keeping with these findings, Clifford et al. in a retrospective study from Switzerland found a threefold excess in carcinomas of the lip, mouth, pharynx and lung in HIV-positive patients, and that no carcinomas from these sites were observed in nonsmokers [4]. UV light exposure is another important risk factor for SCC of the lip [7, 9, 12, 46]. Other potential carcinogenic factors related to oral SCC are marijuana, syphilis, oral sepsis, iron deficiency, and oral candidiasis.

## 5. Mucosal Squamous Cell Carcinoma

SCC of the head and neck comprises a heterogenous group of neoplasms arising from the mucosa of the oral cavity, oropharynx, hypopharynx, larynx, and other sites. The most commonly reported sites for SCC include the oropharynx, conjunctiva, tonsil, and larynx (see Table 1), which is consistent with other studies [27, 38, 50, 51]. Interestingly, a study from Kenya described an 8% prevalence of conjunctival SCC in patients with HIV/AIDS [51]. A number of epidemiological studies have identified an increased risk of SCC of the larynx, oral cavity, oropharynx, lip, salivary gland, and conjunctiva in HIV-positive patients (see Table 2) [7, 10, 12, 14, 16, 21, 26, 27, 50]. Shebl et al. [14] demonstrated increased rates of HIV-related SCC of the salivary gland (SIR 4.9, 95% CI 2.5–8.6). It must be noted, however, that many so-called SCC of the salivary gland may represent metastases from other head and neck sites. A statistically significant increased risk of oropharyngeal, conjunctival and tonsillar SCC has also been shown in patients with AIDS (Table 2) [7, 9, 10, 12]. As in the general population, SCC of the oral cavity in patients with AIDS may present as an ulcerated or fungating mass or as erythroplakia [10, 20]. Data regarding the incidence and risk of mucosal SCC precursor lesions in patients is limited. However, it is likely that the clinical distinction between benign conditions (e.g., aphthous or infectious ulcers), neoplastic erythroplakia and SCC may be challenging. Most of the affected HIV-positive patients reported to date presented at a younger age and advanced stage at presentation [10, 11, 18, 19, 48]. In general, an overall younger age at presentation has been reported for HIV-associated SCC of the head and neck [10, 11, 18, 19, 48]. One study demonstrated a mean age of 36 years [18].

The histopathologic features of SCCs arising in the head and neck range from well differentiated tumor with obvious squamous differentiation and keratinization to poorly differentiated carcinomas lacking keratinization (see Figure 1). Keratinizing carcinomas are more typical of the oral cavity and larynx, whereas nonkeratinizing morphology is seen more commonly in the oropharynx, the latter of which is associated with HPV (see Figure 2). While several morphologic variants of SCC (e.g., verrucous, basaloid, and spindle cell carcinoma) exist, these have not been documented to have a different incidence in the setting of HIV as compared to the general population. A recent study by McLemore et al. [27] described the presence of multinucleated tumor giant cells in 39 of 40 head and neck SCC arising in patients with HIV/AIDS. This feature has not been previously reported. We reviewed cases of mucosal SCC in HIV-positive patients from our institution and also identified these multinucleated tumor giant cells (see Figure 3). Otherwise, the morphologic features of SCCs in HIV patients are not particularly distinct despite the aggressive clinical behavior in this setting.

SCC of the conjunctiva is far more common among HIV-infected individuals compared to HIV-negative persons. A dramatic increase in conjunctival SCC has been reported in sub-Saharan Africa as well as North America [12, 52]. The lower incidence in Europe is believed to be due to the lower solar UV exposure associated with higher latitudes. HIV-related conjunctival squamous lesions range from intraepithelial dysplasia, to carcinoma in situ and invasive SCC. Conjunctival SCC can be seen in relatively young HIV-positive patients and these cancers may be aggressive. Patients can present with eye irritation, erythema, plaque or tumor nodule. SCC of the conjunctiva also has a high propensity for local invasion into the orbit, and occasionally distant metastases may occur. The most common site of origin is the limbus or transition zone of the eye. A case report described conjunctival SCC arising in a 38-year-old woman that although it was focally keratinized, her carcinoma was unusual in that it demonstrated multifocality [51]. In a hospital-based cross-sectional study from Kenya, Chisi et al. [53] noted the following prevalence of histologic patterns of conjunctival SCC in patients with HIV/AIDS: 47% of cases were poorly differentiated, 28% moderately differentiated, 3% were well differentiated and the remainder of these lesions were in situ [53].

Localized SCC is managed with surgery and/or radiation therapy depending on the anatomic subsite. For more extensive or recurrent lesions systemic or targeted chemotherapy may be considered. Treatment complications such as secondary candidiasis and oral mucositis were more common and severe in HIV-positive patients [16, 54, 55] and the outcome of these patients was significantly worse [56]. However, Kao et al. showed that HIV-positive patients could still tolerate radiation therapy [57]. HAART therapy has not altered the incidence of SCC of the oropharynx and other head and neck sites [4, 10, 16, 58, 59].

## 6. Salivary-Type Carcinomas

Some studies [6, 14], but not all [13], have shown that patients with HIV are at increased risk of developing salivary gland malignancies (see Table 2). Among salivary gland malignancies, the risk of common histologic subtypes seen in the general population such as mucoepidermoid carcinoma, adenoid cystic carcinoma and adenocarcinoma, was not elevated among AIDS patients [14]. However, for LEC and SCC of the salivary gland, the risk was greatly increased in patients with AIDS (SIR 39, 95% CI 16.0–81.0 and SIR 4.9, 95% CI 2.5–8.6 resp.) compared to the general population [14].

The cancer risk for patients with HIV was greatest with LEC. However, a significant risk was also determined for SCC of the salivary gland. Whenever a diagnosis of primary SCC of the salivary gland is considered, it is crucial to rule out a metastatic process from another more common head and neck site to a lymph node within or adjacent to the salivary gland [60]. Coincidentally, the parotid gland in which numerous intraparotid lymph nodes can be found is the most commonly reported site of the so-called primary SCCs of the salivary gland. Histologically, the vast majority of SCC in the salivary gland tend to be high-grade and keratinizing [60]. Unique histologic features of salivary gland carcinoma in patients infected with HIV have not been described.

For patients with HIV, the greatest risk for salivary gland carcinoma was determined to be the LEC subtype [14]. The WHO [60] defines LEC of the salivary gland as an undifferentiated carcinoma accompanied by a prominent non-neoplastic lymphoplasmacytic infiltrate. It comprises less than 1% of all salivary gland tumors arising in the general population and is most common in Inuit (Eskimo) and Asian populations. EBV is associated with almost 100% of LEC cases from endemic areas however, it is usually absent in salivary gland LEC from nonendemic areas. EBV isolated from salivary gland LEC from endemic areas reveals the presence of a clonal episomal form of the virus. LEC of the salivary gland develops as a result of a complex interaction of ethnic, geographic and viral factors [60]. LEC tends to arise de novo however it can rarely arise from lymphoepithelial sialadenitis. Morphologically, salivary gland LEC is indistinguishable from the more common nasopharyngeal carcinoma (NPC). As with SCC in the salivary gland, the vast majority of LEC are diagnosed within the parotid gland [60].

Histologically, the malignant cells of LEC are arranged in infiltrative sheets and islands with abundant lymphoid stroma consisting of polymorphous lymphocytes and plasma cells (see Figure 4). Tumor cells have indistinct borders with pale eosinophilic cytoplasm and variable vesicular nuclei with prominent nucleoli. Apart from NPC, other malignant entities to consider in the differentiation include malignant lymphoma and undifferentiated carcinoma. Mitoses are common in LEC and so are necrotic foci. Focal squamous differentiation can be seen. Less common features include noncaseating granulomas, multinucleated giant cells, amyloid and cystic structures. Perineural and angiolymphatic invasion may be seen. The tumor cells are immunoreactive for pancytokeratin and epithelial membrane antigen (EMA). Salivary gland LEC arising in endemic areas typically demonstrate positivity for EBER (see Figure 4).

Both LEC and SCC of the salivary gland are typically treated with surgery and radiation therapy for localized disease. Systemic chemotherapy may be utilized for widespread or metastatic disease. Survival is based on stage of disease, with lower stages demonstrating greater 5-year survival. However, as discussed above, patients with profound immunosuppression will likely poorly tolerate surgery, radiation and/or chemotherapy.

## 7. Nasopharyngeal Carcinoma

In one of the earlier studies, no increased risk of NPC was seen in patients with AIDS in the USA [15]. In a total of 50,050 patients with AIDS, only 4 NPC were diagnosed. Later studies such as that reported by Frisch et al. did demonstrate an increased risk of NPC in AIDS patients (SIR 2.6, 95% CI 1.8–3.8) [9]. The most recent comprehensive study by Shebl et al. also demonstrated an increased risk for NPC for all histologic subtypes (SIR 2.0, 95% CI 1.4–2.7) [14]. The highest SIR in their paper was calculated for nonkeratinizing SCC of the nasopharynx (SIR 2.8, 95% CI 0.9–6.6), followed by nonkeratinizing carcinoma of the nasopharynx (SIR 2.4, 95% CI 1.2–4.4), keratinizing NPC (SIR 2.4, 95% CI 1.5–3.7), LEC of the nasopharynx (SIR 2.1, 95% CI 0.7–4.9) and other subtypes (SIR 1.1, 95% CI 0.5–2.3) (see Table 2). Other studies, but not all, have also demonstrated an increased risk of NPC, and the variability among these studies most likely relates to the rarity of this neoplasm in all populations [6, 11, 13, 16, 18].

The WHO defines NPC as a carcinoma arising in the nasopharyngeal mucosa that shows light microscopic or ultrastructural evidence of squamous differentiation. It encompasses keratinizing SCC, nonkeratinizing carcinoma (differentiated or undifferentiated) and basaloid SCC. Adenocarcinoma and salivary-gland-type carcinoma are excluded [62]. The most common site of origin is the lateral wall of the nasopharynx, followed by the superior posterior wall [62]. The histopathologic features (see Figure 5) depend on the histologic subtype but should demonstrate evidence of squamous differentiation either by light or electron microscopy. Close to 100% of patients with nonkeratinizing NPC demonstrate positivity for EBV, whereas keratinizing SCC or NPC demonstrates more conflicting results. These tumors are immunoreactive for pancytokeratins (AE1/AE3) and high-molecular weight cytokeratins (cytokeratin 5/6, 34*β*E12) [62]. 

Radiation therapy is the treatment of choice for NPC, albeit that a greater incidence of treatment related morbidities has been reported in patients with HIV infection [16, 54, 55]. As expected, outcome and prognosis are directly related to the stage of carcinoma, with lower stages having a much better outcome.

## 8. Merkel Cell Carcinoma

MCC is a rare neuroendocrine carcinoma of the skin most commonly occurring in elderly men. It is very aggressive with a high frequency of local recurrence and metastases. In immunocompetent individuals, MCC tends to arise in sun-exposed areas, with approximately 50% arising in the head and neck region, especially the periorbital areas [63]. A recent development in the understanding of the pathogenesis of MCC is the discovery of the MCV [41] and there is evidence that conditions causing immunosuppression, including HIV, are important risk factors [64]. Engels et al. calculated a relative risk of 13.4 (95% CI 4.9–29.1) of developing MCC in patients with HIV/AIDS compared to the general population [64]. Primary MCC may also arise in non-cutaneous sites in HIV-positive patients, such as intraparotid lymph nodes [65].

The histologic features of MCC in immunocompromised and immunocompetent are identical, with hypercellular areas composed of “small blue cells” with indistinct cytoplasmic borders, hyperchromatic nuclei with indistinct nucleoli and numerous mitotic and apoptotic bodies scattered throughout the tumor (see Figure 6). Angiolymphatic invasion and surface ulceration may be seen [63]. MCC must be distinguished from other small round blue cell tumors such as small cell carcinoma of the lung and lymphoma. MCC demonstrates immunoreactivity for both neuroendocrine markers (neuron specific enolase, synaptophysin and chromogranin) and cytokeratins (cytokeratin 20 and CAM5.2) (see Figure 6). Paranuclear dot-like positivity with cytokeratin 20 is useful diagnostic feature (see Figure 6). MCC is negative for TTF-1, cytokeratin 7 and LCA which help to distinguish this neuroendocrine tumor from small cell carcinoma of the lung and lymphoma. Many cases of MCC may demonstrate CD117 (c-kit) positivity, however this has not been associated with improved outcome [63, 66]. Thus far, no c-kit-activating mutations have been identified [66].

In a recent review article, Izikson et al. [61] reviewed the clinical characteristics of 11 HIV-positive patients with MCC identified from a literature review, along with 3 additional new cases. Unlike MCC sites in immunocompetent individuals which tends to arise in sun-exposed areas, MCC sites were much more diverse and in non-sun exposed areas, suggesting that UV radiation may be less important in the pathogenesis of MCC in immunocompromised HIV-positive individuals. Of the 14 cases reviewed, 5 patients were diagnosed with MCC of the head and neck region (see Table 3). Sites were MCC was documented included the nose, forehead, ear, cheek and scalp. The average age at diagnosis for all 14 cases was 49 years and for the 5 cases arising in the head and neck, the average age was 46.4 years, both much younger than the average age of 69 years seen in immunocompetent individuals [61]. The range for CD4 count was 63–329 cells/*μ*L and the HIV viral load was undetectable to 187,000 copies/mL in some patients (see Table 3). There does not appear to be a relationship between CD4 cell count and HIV viral load with regard to MCC. All 5 patients received HAART prior to, or in one case following the diagnosis of MCC. The lesions in all 5 patients were surgically excised and some received additional radiation and/or chemotherapy. Their survival ranged from 9–24 months.

## 9. Conclusion

As HIV-positive patients live longer with chronic HIV infection we can anticipate an increase in NADC-like head and neck carcinoma. The head and neck carcinomas reviewed here not only demonstrate an increased risk in HIV-positive patients, but all have in common a known oncogenic viral association. It is well established that virally induced neoplasms occur with increased frequency in immunosuppressed individuals. Studies comparing cancer in other immunocompromised populations, such as transplant recipients, to patients infected with HIV may allow us to better determine which of these carcinomas are truly related to immune deficiency. However, larger cohort studies are required to fully investigate the risks of NADC in patients with HIV infection. The younger age at presentation mandates early screening for carcinomas arising in the head and neck of HIV-positive patients. However, clinical staging of a detected carcinoma poses a challenge since lymph node enlargement in the head and neck is common among HIV-positive patients due to a variety of other reasons.

Further investigations are required to explore the pathogenesis, biology and management in HIV-positive patients with head and neck carcinomas. management of patients with AIDS and head and neck cancer is particularly difficult given that many of these patients may not tolerate chemotherapy or radiation therapy and may also have a greater surgical complication rate [16, 54]. However, since the introduction of HAART, patients with advanced AIDS are becoming a minority and as a result of improved immunity with HAART, there are increased therapeutic options for infected individuals with cancer. There is little information regarding the impact of HAART on SCC of the oropharynx and other head and neck carcinomas. Based upon available data, however, it appears that HAART has not altered the incidence of head and neck carcinomas in HIV-positive patients as is seen with KS [4, 10, 16, 58–60, 62].

## Figures and Tables

**Figure 1:** (a) and (b) Squamous cell carcinoma in situ of the conjunctiva in a 43-year-old HIV-positive man. ((a) hematoxylin & eosin (H&E) stain, 100x magnification; (b) H&E stain, 400x magnification). (c) and (d) Ulcerated (c) invasive moderately differentiated squamous cell carcinoma of the tongue and infiltrating among skeletal muscle bands (d) in a 54-year-old HIV-positive man ((c) H&E stain, 100x magnification; (d) H&E stain, 200x magnification).

**Figure 2:** Detection of HPV by immunohistochemistry for p16 ((a) 400x magnification) and HPV in situ hybridization ((b) 400x magnification) in a nonkeratinizing squamous cell carcinoma of the tonsil. Note the strong diffuse nuclear and cytoplasmic staining with p16 immunohistochemical stain (a) and the focal nuclear dot positivity with HPV in situ hybridization, confirming the presence of HPV within the tumor.

**Figure 3:** Example of the multinucleated tumor giant cells in mucosal squamous cell carcinoma arising in the tongue (a) of a 48 year old HIV-positive man, in the tongue (b) of a 54-year-old HIV-positive man and in the oral cavity (c, d) of a 44-year-old HIV-positive man and, similar to the findings of McLemore et al. [27] ((a)–(d) H&E stain, 400x magnification).

**Figure 4:** Lymphoepithelial carcinoma of the parotid gland. (a) Medium power view demonstrating the association between the high grade neoplasm and the parotid acini (H&E stain, 100x magnification). (b) High power view showing the highly atypical epithelial cells with irregular vesicular nuclei and prominent nucleoli (H&E stain, 400x magnification). (c) A cytokeratin AE1 and AE3 highlighting the high grade epithelial cells (200x magnification). (d) EBER in situ hybridization demonstrating strong diffuse nuclear reactivity. Image courtesy of Dr. E. Leon Barnes (400x magnification).

**Figure 5:** (a) Medium-power view of a nasopharyngeal carcinoma, nonkeratinizing, undifferentiated type (H&E stain, 200x magnification). (b) High-power view demonstrating the high-grade malignant cells with indistinct cytoplasmic borders, irregular nuclei with prominent nucleoli (H&E stain, 400x magnification).

**Figure 6:** (a) Low-power view of Merkel cell carcinoma arising in a transplant patient. Note the hypercellular proliferation of small blue cells within the dermis (H&E stain, 40x magnification). (b) A cytokeratin stain (CAM5.2) demonstrating strong diffuse cytoplasmic staining (400x magnification). (c) Perinuclear positivity is seen with cytokeratin 20 (400x magnification). (d) Synaptophysin demonstrates diffuse cytoplasmic staining.

**Table 1:** Sites of confirmed mucosal SCC in The head and neck in patients with HIV/AIDS in articles reviewed.

Site	Number of cases	Reference
Oropharynx	68	[10, 27]
Conjunctiva	65	[7, 9, 12, 38, 39]
Tonsil	29	[9]
Larynx	18	[8, 27]
Oral Cavity	14	[16, 18, 27]
Lip	13	[16]

**Table 2:** Incidence of head and neck carcinomas arising in patients with HIV and AIDS.

Ref #	Year	Country	# patients	# Cases	Cancer site (Subtype)	SIRs or RR (95% CI)	HIV/AIDS
[4]	2005	Switzerland	7304	11	1 Lip, 4 tongue, 4 mouth, 1 pharynx, 1 NPC (?)	**SIR = 4.1 (2.1–7.4)**	not specified

[6]	1999	S. Europe	5281	2	SG (?)	**SIR = 33.6 (3.2–123.5)**	AIDS
				1	NPC	SIR = 10.3 (0.0–58.8)	AIDS

[7]	2006	Uganda	12,607	3	Thyroid	**SIR = 5.7 (1.1–16.0)**	Not specified
				6	Conjunctiva (SCC)	**SIR = 4.0 (1.5–8.7)**	Not specified

[15]	1996	USA	50,050	4	NPC (2 SCC + 2 LEC)	RR = 2.4 (0.7–6.2)	AIDS

[8]	2002	Australia	8118	6	Lip (SCC)	SIR = ~6 (~2–9.5)*	HIV
			8118	6	Lip (SCC)	SIR = ~6.9 (~1.8–9.6)*	HIV
			7061	4	Lip (SCC)	SIR = ~3.0 (0.8–8.1)*	HIV
			2112	3	Lip (SCC)	SIR = ~9.0 (~3.0–>10)*	AIDS

[16]	2004	UK	8640	7	2 NPC; 3 oral cavity (SCC) 2 larynx (SCC)	SIR = 1.66 (0.67–3.42)	2 (AIDS); 5 (HIV)

[9]	2000	USA	309,365	29	Tonsil (SCC)	**RR = 2.6 (1.8–3.8)**	HIV/AIDS
				7	Conjunctiva (SCC)	**RR = 14.6 (5.8–30.0) **	

[17]	2003	Scotland	2574	1	H&N (unspecified, not KS)	SIR = 1.6 (0.04–8.8)	Unknown

[10]	2009	USA	499,230	59	Oropharynx (SCC)	**SIR = 1.6 (1.2 to 2.1)**	AIDS

[11]	2005	England	33,190	6	Oral (?)	SIR = 1.1 (0.4–2.3)	HIV
				4	NPC (?)	**SIR = 5.0 (1.4–12.8)**	HIV
				1	Nasal Cavity (?)	SIR = 1.7 (0.04–9.4)	HIV
				5	Larynx (?)	SIR = 2.0 (0.7–4.8)	HIV
			12126	5	Oral (?)	**SIR = 3.8 (1.2–8.8)**	AIDS
				1	NPC (?)	SIR = 5.8 (0.1–32.5)	AIDS
				1	Nasal Cavity (?)	SIR = 7.9 (0.2–44.0)	AIDS
				2	Larynx (?)	SIR = 3.2 (0.4–11.6)	AIDS

[12]	2008	USA	491,048	15	Conjunctiva (SCC)	**SIR = 12.2 (6.8–20.2)**	AIDS

[13]	2002	Australia	13,067	10	Lip (?)	**SIR = 2.26 (1.08–4.16)**	Not specified
				2	Tongue (?)	SIR = 1.66 (0.20–5.99)	Not specified
				2	SG (?)	SIR = 3.88 (0.47–14.0)	Not specified
				2	Nasopharynx (?)	SIR = 2.74 (0.33–9.89)	Not specified
				1	Nose/sinuses/ear (?)	SIR = 2.97 (0.08–16.5)	Not specified
				1	Larynx (?)	SIR = 0.60 (0.02–3.34)	Not specified
				1	Eye (?)	SIR = 1.73 (0.04–9.64)	Not specified
				1	Thyroid (?)	SIR = 0.56 (0.01–3.12)	Not specified

[14]	2009	USA	519,934	43	SG (All types)	**SIR = 1.8 (1.3–2.4)**	AIDS
				12	SG (SCC)	**SIR = 4.9 (2.5–8.6)**	AIDS
				7	SG (LEC)	**SIR = 39 (16–81)**	AIDS
				6	SG (Acinar cell ca)	SIR = 1.9 (0.7–4.1)	AIDS
				5	SG (MEC)	SIR = 0.6 (0.2–1.5)	AIDS
				2	SG (Adenoid Cystic Ca)	SIR = 0.6 (0.1–2.0)	AIDS
				2	SG (Adenoca)	SIR = 0.7 (0.1–2.5)	AIDS
				39	NPC (All types)	**SIR = 2.0 (1.4–2.7)**	AIDS
				22	NPC (Ker SCC)	**SIR = 2.4 (1.5–3.7)**	AIDS
				10	NPC (NK Carc)	**SIR = 2.4 (1.2–4.4)**	AIDS
				5	NPC (LEC)	SIR = 2.1 (0.7–4.9)	AIDS
				5	NPC (NK SCC)	SIR = 2.8 (0.9–6.6)	AIDS
				7	NPC (Other/?)	SIR = 1.1 (0.5–2.3)	AIDS

Bold values indicate cancer sites where the 95% confidence interval does not include one.

SIR: standardized incidence ratio, RR: relative risk, SG: salivary gland, SCC: squamous cell carcinoma, NK: nonkeratinizing, NPC: nasopharyngeal carcinoma, H&N: head and neck, Ker: keratinizing, LEC: lymphoepithelial carcinoma, Adenoca: Adenocarcinoma.

**Table 3:** Merkel cell carcinoma in head and neck sites of HIV positive patients (reproduced from Izikson et al. [61]).

Sex	Race	Age (years)	Site	HIV Dx to MCC (years)	CD4 (cells/*μ*L)	Viral load (copies/mL)	Treatment	On HAART	Survival (months)
M	NA	60	Nose	NA	329 (2 yrs after Dx)	NA	Mohs XRt	Yes	24
M	NA	63	Forehead	12	232	Undetectable	Mohs	Yes	NA
F	African black	36	Left ear	NA	63	24,000	WLE	Yes	>9
F	African black albino	25	Right cheek	NA	332	187,000	Chemo, XRt, WLE	Yes (after Dx)	12
M	Caucasian	48	Scalp	12	Normal	Undetectable	WLE, XRt	Yes	>12

Dx: diagnosis, XRt: radiation therapy, NA: not available, Chemo.: chemotherapy, WLE: wide local excision.
